# The Skill Training of Reading Music in the Teaching of Solfeggio and Ear Training in the New Media Environment

This article has been retracted.

**DOI:** 10.1155/2022/8209861

**Published:** 2022-03-19

**Authors:** Lin Wang

**Affiliations:** School of Music, Northwest Normal University, Lanzhou, 10736 Gansu, China

## Abstract

Culture is a powerful spiritual force rooted in the hearts of the Chinese people and guides the direction of the Chinese people. Sight singing and ear training are playing an increasingly important role as an important means of music teaching. The article is aimed at studying the latest application progress of music reading skills in audiovisual ear training in the new media environment. This paper proposes the interactive application of music reading skills that integrate new media to realize the interactive communication between man and machine. The experimental results of this paper show that new media can make greater use of the advantages of music reading skills, enhance students' musical sensitivity by 20%, and realize musical interaction.

## 1. Introduction

The society continues to progress and develop; people's demand for beauty is further improved, and music and other artistic activities are becoming more and more sought after by people. Music is the art of listening, and good musical hearing is the basis for appreciating and creating music. As a basic subject of music, sight singing and ear training have been recognized by more and more music experts and scholars for their importance. It has been continuously developed and updated in music teaching. Learning solfeggio and ear training can enhance students' aesthetic and perception of music and spread the cultural connotation of music. In the new era, when the needs of spiritual civilization cannot effectively meet the wishes of the masses, it is undoubtedly an urgent task to strengthen the education of sight singing and ear training and cultivate more music talents. Sight singing and ear training are based on two major parts: sight singing and ear training. Among them, the foundation of sight singing is singing; reading score is the focus; the foundation of ear training is listening, and the rhythm is the focus. The new media technology of the new era has opened up new channels for sight singing and ear training. For the training of reading music, experts and scholars at home and abroad have achieved some results after long-term research. Maturi and Sheridan explore the ability to locate music reading knowledge and compare the eye movements of 30 professional musicians and 30 nonmusicians when completing a visual search task that requires them and match a part of a complex piano score with the same corresponding part in a larger score. The experiment allows search templates and arrays to be presented simultaneously for visual comparison in each experiment of the experiment. It is concluded that experts use domain-specific knowledge in the form of “blocks” and “templates” to obtain accurate representation templates for highly complex searches [1]. Aycan observed whether the pronunciation syllables formed a rhythmic structure in the sight singing and ear training. He checked the adaptation of Bona's (rhythmic pronunciation practice) vocal practice in the course. In conclusion, Bona practice occupies an important position in sight singing and ear training. The correct intonation or tone can be obtained through the principle of correct vocalization, using the strength of consonants and voicing syllables by affecting the strength, duration, and tone strength of the speech. Reading notes according to intensity and performing breathing exercises are very helpful to pronounce consonants and find tones [2]. Bennett introduced the application of Apple iOS in music production and his understanding of the upward trend of analog systems. He set chapters in different editions of textbooks on recording and music production as required reading for vocational training courses and university degrees. He believes that related content and symbiosis with standard recording and production courses are the two key advantages of this book, but its overall accessibility and crucially its rhythm set this textbook apart from similar titles [3]. Slater et al. study the factors that influence musicians' cognitive and sensory processing enhancement and investigate the influence of major musical instruments on musicians' professional knowledge signatures by evaluating three groups of young people. Assuming that the main instrument will produce selective enhancements that reflect the most significant acoustic characteristics of the instrument, regardless of the instrument, the cognitive function will be enhanced. Consistent with the hypothesis, compared with nonmusicians, percussionists show more accurate coding of rapidly changing voice acoustic characteristics, while vocalists have better frequency discrimination and stronger speech overtone coding than nonmusicians. Compared with improvisation, specialization has no obvious advantage in sight reading [4]. The Jain and Nataraja's study evaluated the effects of fatigue on the working memory and hearing of trained instrument musicians. 26 well-trained instrument musicians and 25 nonmusicians were found to participate in the study. The effects of fatigue are assessed by performing working memory and auditory perception tests under pre- and postfatigue conditions. The conclusion is that the advantage of music training on working memory may be weakened by fatigue. Therefore, musicians should take measures to reduce fatigue [5]. Kalathottukaren et al.'s study compares the prosody perception and production ability of children with hearing loss and children with normal hearing. They investigate the influence of age, listening level, and musicality on the perception of rhythm. Compared with the control group, all PEPS-C subtests and total scores of children with hearing loss were significantly reduced (*p* < 0.05). In conclusion, children with hearing loss between the ages of 7 and 12 have significant difficulties in understanding different aspects of prosody and are rated as having more atypical prosody than the control group in general. These findings indicate that clinical evaluation and speech-language therapy services for children with hearing loss should be expanded to address prosody difficulties [6]. The article studies the reading skills in the teaching of solfeggio and ear training. Through interactive learning of new media, the content of reading training is optimized, and the efficiency of reading training is improved. To help students better master the training of reading scores, integrate the teaching of sight singing and ear training faster, and realize the improvement of musical skills.

## 2. Solfeggio and Ear Training and New Media

### 2.1. Solfeggio and Ear Training

Sight singing and ear training are basic subjects, which require high technical requirements and require the comprehensive development of students [7]. As shown in Figure 1, solfeggio ear training includes two aspects: first, sight singing training; to get the score, students must first be able to analyze the content of the score and then through the score to develop sight singing exercises to improve the ability to read and sing. The second is ear training, as the name suggests is to exercise hearing. Students should grasp the changes in the rhythm of music, have a strong sense of sound, and have a good musical hearing ability. Sight singing and ear training are basic subjects for all music lovers and learners, and such play an important role in the history of music education [8].

The prerequisite of sight singing training is to understand music. To understand music, knowing how to read sheet music is very important. Sheet music is the carrier of the dissemination of music text, which can promote communication and inheritance to a certain extent. Therefore, the first step in understanding music, appreciating music, and creating music is to learn to read and understand music scores. Music reading training is a very important part of the teaching of sight singing and ear training. It is more than just reading and reading scores in a literal sense, but more deeply is to understand the changing laws of music through music scores and how to play and show this musical melody. Music reading training is a manifestation of students' musical literacy. The premise of developing musical reading training is to sing a roll call and express music quickly and accurately. The key to auditory training lies in the cultivation of inner voice. It is the foundation of all music-related activities and is essential for improving music listening ability. Inner voice and notation reading training promote each other and complement each other. In the process of reading scores, the inner hearing must be able to control the sound to express the image of the music, so as to cultivate the perception of music rhythm, melody, structure, and so on. In the process of training inner hearing, inner hearing can cultivate the foresight and imagination of music reading, enhance music vitality, better control sound, and realize the cultivation of musical expression and perception.

### 2.2. Solfeggio and Ear Training Skills

#### 2.2.1. Methods of Sight Singing Training

1. Training of Interval

First, the interval can be classified into melody interval and sound interval. The difference is that the two tones of the former are different at the same time and sound sequentially; in the latter, the two tones are sounded at the same time. As shown in Table 1, the author needs to understand the sound effects and interval colors of various intervals [9].

From the above table, the author can see the degree of harmony and color of different intervals within an octave. In addition, there is also a difference between large and small intervals. In summary, the large intervals are relatively active and bright, while the small intervals are soft and dim. Intervals need to be practiced on the basis of this theory. In Figure 2 (1), the beginning of the score is a three-degree jump. When student practice, student r can use the bridge method to sing, mi-sol, teacher can sing mi, fa, sol first. Because it is a big dotted rhythm, it is not as regular as quarter notes. Therefore, when student practice sight singing, teacher sing mi as one beat, and fa and sol form a double-eight rhythm pattern. After establishing the correct concept of pitch and value, you can directly perform three-degree singing. When performing third-degree singing directly, the bridge in the middle should sing silently, that is, sing silently and attentively. In fact, this is also a kind of training of inner music hearing through interval bypass training.

In Figure 2 (2), the music is a good piece of music for interval training. It is an exercise for transposition of the third and the sixth degree in the interval. Due to changes in the score, the original single-tone music has become two-tone music. At this time, the teacher can analyze the music score for the students first, teach the knowledge of music theory, and then, demonstrate for the students. Let students listen and observe the changes in finger distance and the color of the sound and finally express their feelings after listening in their own words.

(2) Chord Practice

A chord is composed of more than three (including three) tones of different pitches, combined according to a certain rule. Compared with the interval, it is more difficult to listen to the chords. The chord structure mainly includes the second, third, and fourth intervals. For the training of chords, student mainly adopt the training of hearing and feeling the color of the chords [10]. In the music score, when there are a lot of chords, the teacher selects different chords and makes a chord connection, so that students can play and sing while playing. Sing from the bass mode to the treble and then sing back to the bass from the treble mode. Through this practice of singing the chords, the nature of the chords can be distinguished. Use your fingers to feel the distance change of the sound when playing, reducing the difficulty of the learner to play the whole piece of music. Use your ears to feel the changes in the color of the chords, and experience the sense of color of the chords. First, analyze the harmony colors and sound effects of various chords (take triads and sevenths as examples), as shown in Table 2. The major triad has a broad and bright color because the root to third tone is the major third; minor triads are soft and dim in color because the roots to thirds are minor thirds; since the structure of diminished triads is composed of minor thirds, it gives people a sense of tension and oppression in the auditory sense; the structure of the augmented triad is composed of two major thirds, so it gives a sense of expansion and a stronger sense of disharmony.

The training of staff reading ability can be divided into five steps [11], as shown in Figure 3.

(3) Music Reading Training
(1) Sing only the pitch. After students get a staff and determine the key, they can only sing regardless of the rhythm, so as to train the sense of pitch

The distance between the adjacent two notes of this sight singing practice is relatively close. In our first training, teacher can reserve the tone first, remove the rhythm, and practice the pitch and interval first, as shown in Figure 4 for sight singing. In the sight singing pitch, students can use the combination of fixed and first tune to practice. In the sight singing pitch, students can use the combination of fixed and first tune to practice. Firstly, train the sense of pitch through the fixed roll call; then, train the sense of mode and pitch through the first roll call. The key signature of the example score is two sharps, which belong to the D house system tone. The first F note should be sung with mi in the D palace system tune with the first tune roll name, and so on.

(2) Look at the score and sing the rhythm. Singing the rhythm is the second step. In this training process, remove the pitch, keep the rhythm, and sing the rhythm completely with “Da” while tapping. If you are worried about the inaccuracy and unevenness of the beat, you can use the metronome to fix the beat. First, slow down and sing each rhythm smoothly and clearly, then gradually increase the speed
(3) Combination of intonation and rhythm. In a music score, pitch and rhythm are the foundation. After passing the previous basic training, on the basis of ensuring the intonation, adding the rhythm pattern to practice, the recognition of a staff is basically completed
(4) Music emoji. Of course, to complete a sight singing with a staff, it is not enough to focus on the basic intonation rhythm. In addition to the intonation rhythm, there will also be some musical emoticons in the score, such as crescendo, fading, crescendo, speed, speed, and other emoticons

As shown in Figure 5, this score is marked with a crescendo mark, which requires us to perform a comparison of strengths and weaknesses while completing the basic scores to show the emotion and color of the music.

(5) Musical breathing. Finally, student must pay attention to the breathing of the music, and the phrase segmentation, so as to make the music more complete

As shown in Figure 6, the melody has a phrase every two bars. When singing the score, you should pay attention to breathe every two bars to make the music flow more contagious.

#### 2.2.2. Methods of Ear Training

1. Beat Training

Rhythm is the skeleton of the melody, so the beat is the pulse of the melody [12]. Rhythm training is first to feel the strength and weakness of the rhythm changes. It can be said that beat training is the basis of rhythm training. If you want to feel this law, then the best interpretation is the unit beat represented by quarter notes. Because this unit beat can show two moments of rhythm change, namely, the stronger moment and the weaker moment, and the cycle of strong and weak alternates, this allows us to easily close to the beat of the music.

Figure 7 (1) is a piece of music in four or four beats. The four or four shots are like shooting a ball. The strong shots are shot with the right hand and the weak shots are shot with the left hand. Figure 7 (2) is a piece of music in four or three beats. Four and three beats are strong, weak, and weak. The impression of the first shot is a sense of sinking, the impression of the second shot is that the music has an upward trend, and the third shot makes people feel like swinging on a swing.

(2) Rhythm Training

Rhythm can be interpreted as a sequence of lengths that vary with the time value of the note [13]. It is a complete way of expression, specifically expressed in the intensity and length of the sound. In rhythm training, we first choose the rhythm of reading aloud. When we encounter a new learning rhythm, we do not need to read aloud in the traditional way of “da, da, da, da,” but use our own closer language to interpret their lifestyle, for example, your name and phrases you just learned to train your rhythm. Under the guidance of the teacher, after the rhythm reading practice, let the students sing the music, tap with their right hand, and sing with emotion. In rhythm training, there are more difficult rhythms, such as fixed tone rhythm, segmented rhythm, triplet, and eighty-three and eighty-six beats. The teacher explains the duration of the sound value to the students, so that the students can really feel the change in the value of the time. For example, when we recite ancient poems, the teacher will read some longer words and some shorter words and compare the differences between different notes in order to learn better.

### 2.3. Theories Related to Sound Propagation

The basis of the speaker's ability to raise the sound is that it expands the sound in different directions as the sound spreads. Its directivity basis is composed of the structure and principle characteristics of the speaker. Directivity diagram, directed frequency response, directivity index, and directivity factor are commonly used measures of speaker directivity [14, 15]. The directivity diagram refers to the construction of a polar coordinate image of the directivity function *G*(*ω*) of the sound source that changes the radiation sound pressure level with the radiation direction. Test the distance by measuring the sound pressure level of the free-field image at different frequencies. According to the definition: the directivity function can be expressed as:

(1) $$\begin{array}{c} G\left(\omega \right)=\frac{S\left(\omega \right)}{S\left(0^{{}^{\circ}}\right)}. \end{array}$$

Among them, *S*(*ω*) is the sound pressure in the *ω* direction under equidistant conditions, and *S*(*O*°) is the sound pressure in the initial direction.

The directivity factor is the ratio of sound intensity, which represents the ratio of the sound intensity of a directional sound source to the sound intensity of a nondirectional sound source at the same power and location, which is

(2) $$\begin{array}{c} Z=\frac{L_{A}}{L_{B}}. \end{array}$$

In the formula, the directivity factor can be expressed by *Z*. The sound intensity of the sound source on the directional sound source can be represented by *L*_*A*_, and the sound intensity of the nondirectional sound source at the same position can be represented by *L*_*B*_.

A common indicator for measuring the directivity of a loudspeaker is the directivity factor *Z* or the directivity index *F*. The relationship between *Z* and F *i*s as follows:

(3) $$\begin{array}{c} F=10\mathrm{lg}Z. \end{array}$$

The pointing frequency response is a set of curves of the frequency response at a specific distance, which deviates from the direction of the reference axis. Based on the linear propagation characteristics of small-amplitude sound waves, small-amplitude sound waves can be superimposed and expressed by wave equations. Suppose *r*_1_ and *r*_2_ are the sound pressures of the two rows of sound waves, and *r* is the sound pressure of the synthesized sound field. According to the sound wave equation, the synthetic sound field *r* must also satisfy the wave dynamic range [16], which is

(4) $$\begin{array}{c} \nabla^{2}r=\frac{1}{d_{0}^{2}}\frac{\partial^{2}r}{\partial t^{2}}. \end{array}$$

On the other hand, sound pressures *r*_1_ and *r*_2_ also satisfy the sound wave equation, namely,

(5) $$\begin{array}{c} \nabla^{2}r_{1}=\frac{1}{d_{0}^{2}}\frac{\partial^{2}r_{1}}{\partial t^{2}}, \end{array}$$

(6) $$\begin{array}{c} \nabla^{2}r_{2}=\frac{1}{d_{0}^{2}}\frac{\partial^{2}r_{2}}{\partial t^{2}}. \end{array}$$

If (5) and (6) are added together, we can get

(7) $$\begin{array}{c} \nabla^{2}\left(r_{1}+r_{2}\right)=\frac{1}{d_{0}^{2}}\frac{\partial^{2}\left(r_{1}+r_{2}\right)}{\partial t^{2}}. \end{array}$$

Based on the acoustic boundary conditions which are also linear, we can get:

(8) $$\begin{array}{c} r=r_{1}+r_{2}. \end{array}$$

The synthesized sound field of the two rows of sound waves is equal to the sum of the sound pressure of each row of sound waves, which conforms to the principle of superposition of sound waves. In the same way, it can be inferred that multiple rows of sound waves conform to the principle of sound wave superposition [17].

The interference phenomenon is a phenomenon caused by the superposition of two rows of sound waves with the same frequency and a certain phase difference [18]. Assume that the two series of sound waves are:

(9) $$\begin{array}{c} r_{1}=r_{1b}\cos\left(\varepsilon t-\delta_{1}\right), \end{array}$$

(10) $$\begin{array}{c} r_{2}=r_{2b}\cos\left(\varepsilon t-\delta_{2}\right). \end{array}$$

Suppose *δ* = *δ*_2_ − *δ*_1_ is the phase difference of the two series of sound waves and does not change with time. Based on the principle of superposition, the sound pressure of the synthesized sound field is

(11) $$\begin{array}{c} r=r_{1}+r_{2}=r_{1b}\cos\left(\varepsilon t-\delta_{1}\right)+r_{2b}\cos\left(\varepsilon t-\delta_{2}\right), \end{array}$$

(12) $$\begin{array}{c} r=r_{b}\cos\left(\varepsilon t-\delta \right), \end{array}$$

where

(13) $$\begin{array}{c} r_{b}^{2}=r_{1b}^{2}+r_{2b}^{2}+2r_{1b}r_{2b}\cos\left(\delta_{2}-\delta_{1}\right), \end{array}$$

(14) $$\begin{array}{c} \delta =\arctan\frac{r_{1b}\sin\delta_{1}+r_{2b}\sin\delta_{2}}{r_{1a}\cos\delta_{1}+r_{2a}\cos\delta_{2}}. \end{array}$$

The formula shows that although the synthetic sound pressure is sound vibration of the same frequency, there is no correlation between the synthetic sound pressure amplitude and the sum of the sound pressure amplitudes of the two sound waves, but there is a correlation with the phase difference *δ*.

The average energy density in the sound field can be expressed by the square of the sound pressure amplitude. Then, the average energy density of the synthesized sound pressure can be expressed as:

(15) $$\begin{array}{c} m=m_{1}+m_{2}+\frac{r_{1b}r_{2b}}{\rho_{0}d_{0}^{2}}\cos\delta . \end{array}$$

In the formula, *m*_1_ and *m*_2_ are the average energy densities of *r*_1_ and *r*_2_, respectively, indicating that there is a correlation between the average energy density and the phase difference *δ*.

If there are *δ* = 0, 2*π*, 4*π*, ⋯ in some positions, it means that the two trains of sound waves always arrive at the same phase, then

(16) $$\begin{array}{c} r_{b}=r_{1b}+r_{2b}, \end{array}$$

(17) $$\begin{array}{c} m=m_{1}+m_{2}+\frac{r_{1b}r_{2b}}{\rho_{0}d_{0}^{2}}. \end{array}$$

If there is a *δ* = ±*π*, ±3*π* ± 5*π* in some other positions, which means that the two rows of sound waves always arrive in opposite phases, then

(18) $$\begin{array}{c} r_{b}=r_{1b}‐r_{2b}, \end{array}$$

(19) $$\begin{array}{c} m=m_{1}+m_{2}‐\frac{r_{1b}r_{2b}}{\rho_{0}d_{0}^{2}}. \end{array}$$

The formula shows that the average energy density is only related to the phase difference of the two sets of sound waves in the superposition field of two sets of sound waves with the same frequency and a certain phase difference.

### 2.4. New Media

New media, or digital media, network media, is the sum of media with communication functions based on information processing computer technology and the Internet [19]. It has three common characteristics: first, it is based on the emergence of digital technology and network technology; the second is to use electronic devices such as computers and mobile phones as the main receiving end; the third is to provide information to users [20]. From the analysis of the definition of new media and the interpretation of the practice of new media communication, we can conclude that new media has four basic characteristics [21]: first, technology. New media is a digital information transmission technology based on the Internet. The development of network and digital technology provides reliable and efficient technical support for new media. This kind of network transmission is faster, more accurate, and smarter in content, and is very different from traditional media in content and form. Second is timeliness. Timeliness is an important criterion for measuring news and news vitality. The new media dilutes the constraints of time and space. As long as the two conditions of digital terminal and network connection are met, information can be received and sent anytime and anywhere, which compared with any other means of communication, it has obvious advantages. Third is interactivity. New media has overturned the one-way communication of traditional media, made the sharing of network information resources more convenient, made news sources and communication trends more diversified, and made communication present a multidirectional communication trend. Fourth, personalization. The emergence of new media has further made up for the shortcomings of traditional media, not only pursue various forms of visual and auditory stimulation but also require more information. New media can provide users with a series of services based on their habits, preferences, and information usage characteristics.

## 3. Reading Music Survey Experiment and Analysis

### 3.1. Experimental Subjects and Experimental Design

Among the first-year students in a music school, two classes with similar grades were randomly selected to start reading training. One class used new media to carry out music reading training, and the other class carried out music reading training according to the traditional model, and the control variables kept other conditions unchanged. After conducting a period of training in reading music, test the results of the two classes, investigate students' feelings, and understand their views on the training in music reading.

### 3.2. Building a New Media Teaching Platform

As shown in Figure 8, instead of the traditional piano blackboard, the new media builds an interactive teaching platform. With the help of projectors, computers, MIDI keyboards, speakers, curtains, and other appliances, and through teaching and learning, human-computer interaction, etc., it increases the perception and understanding of learning music skills and strengthens communication, so as to achieve the purpose of learning in interaction and growth in communication.

### 3.3. Experimental Data Processing

Collect the changes in student performance before and after the experiment; analyze and evaluate the effect of the experiment. Investigate the feelings of students and teachers, understand their opinions on the integration of new media in reading music training, and collect and record relevant information.

### 3.4. Data Analysis

It can be seen from Table 3 that the general situation of the experimental class and the control class are the same. They are all students who have just entered the school for a short period of time, and they have carried out music reading training for about one month, which can compare the effects of music reading training under the new media. There is a difference in the sex ratio between the two groups, but the difference is not big. In general, the data of the experimental group and the control group are consistent.

It can be seen from Figure 9 that after a certain period of training, the student's performance generally rises. On the whole, the pitch and rhythm have improved the most before and after the training, and the special new media's music reading training has a better effect than traditional methods. This may be due to the fact that new media has enriched students' interests through images, audio, video, and other forms of interaction, complementing the weaknesses of the students' foundation and leading to a faster improvement in grades.

It can be seen from Figure 10 that there are also gender differences in music reading training. Women have a better foundation in pitch and rhythm, and men have a better foundation in expression and breathing. After a period of training, all indicators have improved, but overall, men have improved more. It shows that training can better improve performance. At the same time, although expression and breathing have improved, the improvement is relatively low. It may be because breathing and expression are more detailed and controlled, requiring long-term inspections, and short-term training is slower.

It can be seen from Figure 11 that students have a good overall experience of the new media-integrated music reading training. Before training, students are more supportive of new media music reading courses. After feeling the advantages of new media courses, the recognition of students has further improved. Although the proportion is small, we should also see that some students still do not approve of new media reading training. Investigating the reasons, there are reasons why I do not like not only music reading training but also slow performance improvement. This will be further optimized and improved in the future.

It can be seen from Figure 12 that at first, teachers did not approve of the music reading training of new media integration. They feel that traditional methods have sufficient teaching experience and are more suitable for students. Taking the new method rashly may have an impact on student performance. After the implementation of new media-integrated music reading training, students' performance indicators have improved, so teachers have an impression of new media-integrated music reading training. However, there are still teachers who do not recognize the teaching methods of new media. It may be that new media has increased the burden on teachers, and some teachers are not familiar with new media.

## 4. Discussion

Regarding the effect of new media-integrated music reading training, the article designed a controlled experiment to measure the impact of new media-integrated music reading training on students and teachers while ensuring that other factors remain unchanged. In general, the new media-integrated music reading training has a positive impact on students. The rich and interesting new media content helps students increase their interest in learning, and the focused framework helps students check for deficiencies. While the new media trains notation reading skills, it further enhances students' learning information. On the other hand, new media-integrated music reading training also puts forward new requirements for learning equipment and teachers' abilities. In the future, the author expects that with the help of new media, students can develop a sense of sight singing and ear training more quickly, master the skills of reading scores, truly appreciate the beauty of music, and enjoy the beauty of music.

## 5. Conclusions

Based on the new media environment in the teaching of solfeggio and ear training, this paper conducts research on the training of reading music skills and gives a detailed introduction to the teaching skills of solfeggio and ear training. It also illustrates the relative advantages of reading music skills training. Design a control experiment of new media fusion music reading training, which confirmed the advantages of new media in training music reading skills. With the investigation of teachers and students' experience, new media-integrated music reading training will definitely give play to greater advantages to help students grow. But the research also has certain problems: the sample surveyed in article is too small and may not be representative. The research in article only focuses on the improvement of academic performance and lacks investigation in other fields. New media requires supporting equipment, which increases the cost of schools. For teachers, accepting and using new media are a challenge.

## Figures and Tables

**Figure 1:** Schematic diagram of the structure of sight singing and ear training.

**Figure 2:** Schematic diagram of interval training.

**Figure 3:** The structure diagram of reading music training skills.

**Figure 4:** Schematic diagram of interval extraction in music reading.

**Figure 5:** Schematic diagram of expression changes in music reading music.

**Figure 6:** Schematic diagram of breathing pause in music reading.

**Figure 7:** The difference between four or four beats and four or three beats in beat training.

**Figure 8:** Schematic diagram of teaching platform.

**Figure 9:** Comparison of the results of the experimental group and the control group before and after the experiment.

**Figure 10:** Comparison of differences in performance between men and women in music reading training.

**Figure 11:** Survey of students' feelings about new media-integrated music reading training in music reading training.

**Figure 12:** Teachers' feelings about new media-integrated music reading training in music reading training.

**Table 1:** Sound effects and interval colors of various intervals.

Interval	Sound effect	Interval color
Pure one degree, pure octave	Extremely concord	The sound is extremely integrated, but hollow and thin
Pure fourth degree, pure fifth degree	Full concord	The sound is fusion, more pleasing but hollow and thin
Major third, minor third, major sixth, minor sixth	Incomplete concord	The sound is more integrated and rich and full
Major second, minor seventh, increase four degrees, decrease five degrees	Disharmony	The sound is not fused, it is sharper and harsher
Major seventh, minor second	Extremely incongruous	The sound is extremely unmixed, sharp, and harsh

**Table 2:** Analysis of harmony color and sound effect of chord training.

Chord	Harmony color	Sound effect
Major triad and its inversion	Bright and powerful	Concord
Minor triads and their inversions	Soft and dim	
Increased triad and its inversion	Tighten inward	Disharmony
Minus triad and its inversion	Expand outward	
Seventh chord		

**Table 3:** Introduction to experimental class and control class.

	Experimental class	Control class
Female	18	21
Male	12	9
Total	30	30
Age	18	18
Training time	30	30

## Data Availability

All the data used is given in the paper.

## References

[1] Maturi K. S., Sheridan H. (2020). Expertise effects on attention and eye-movement control during visual search: evidence from the domain of music reading. *Attention, Perception, & Psychophysics*.

[2] Aycan K. (2017). Using bona adaptation to improve accent defects as a voice training method. *Eurasian Journal of Educational Research (EJER)*.

[3] Bennett S., Huber D. M. (2018). *Modern Recording Techniques*.

[4] Slater J., Azem A., Nicol T., Swedenborg B., Kraus N. (2017). Variations on the theme of musical expertise: cognitive and sensory processing in percussionists, vocalists and non-musicians. *European Journal of Neuroscience*.

[5] Jain S., Nataraja N. P. (2019). The effect of fatigue on working memory and auditory perceptual abilities in trained musicians. *American Journal of Audiology*.

[6] Kalathottukaren R. T., Purdy S. C., Ballard E. (2017). Prosody perception and production in children with hearing loss and age- and gender-matched controls. *Journal of the American Academy of Audiology*.

[7] Rozgus A. (2019). Technology is pervasive: are you ready?. *Consulting-Specifying Engineer*.

[8] Tavera Romero C. A., Hamilton Ortiz J., Khalaf O. I., Ortega W. M. (2021). Software architecture for planning educational scenarios by applying an agile methodology. *International Journal of Emerging Technologies in Learning*.

[9] Babik D., Singh R., Zhao X., Ford E. W. (2017). What you think and what I think: studying intersubjectivity in knowledge artifacts evaluation. *Information Systems Frontiers*.

[10] Comings J. P., Strucker J., Bell B. (2017). Two reading assessments for youth in alternative basic skills and livelihood skills training programs. *Prospects*.

[11] Xu H. (2019). Analysis on the innovative paths of university campus culture construction under the new media environment. *International Journal of Social Science and Education Research*.

[12] Eagle L., Dahl S. (2018). Product placement in old and new media: examining the evidence for concern. *Journal of Business Ethics*.

[13] Zhou D., Li B. (2017). How the new media impacts rural development in China: an empirical study. *China Agricultural Economic Review*.

[14] Alkhafaji A. A., Sjarif N. N., Shahidan M. A. (2021). Payload capacity scheme for quran text watermarking based on vowels with kashida. *CMC Computer, Materials and Continua*.

[15] Hendrickson B., Rosen D. (2017). Insights into new media use by international students: implications for cross-cultural adaptation theory. *Social Networking*.

[16] Simone N. (2017). *Updating to remain the same: habitual new media*.

[17] Walter B., Schmid R., Delius S. V. (2017). Improving patient information – are the new media already requested? – a questionnaire study at a gastroenterology outpatient clinic. *Zeitschrift für Gastroenterologie*.

[18] Chen C., Cheng L. (2020). African youth languages: new media, performing arts & sociolinguistic development. *Journal of African Languages and Linguistics*.

[19] Hinnosaar M. (2019). Gender inequality in new media: evidence from Wikipedia. *Journal of Economic Behavior & Organization*.

[20] Zhao H., Chen P.-L., Khan S., Khalafe O. I. (2021). Research on the optimization of the management process on internet of things (Iot) for electronic market. *The Electronic Library*.

[21] Editor J. L. R. G., Editor-In-Chief W. Z. S. (2017). Old journal, new media. *Asian Journal of Anesthesiology*.

